The article "Phytochemical Analysis, Antioxidant, Antimicrobial, and Anti-Swarming Properties of Hibiscus sabdariffa L. Calyx Extracts: In Vitro and In Silico Modelling Approaches" was published in 2022. Journal: Evid Based Complement Alternat Med.

# Phytochemical Analysis, Antioxidant, Antimicrobial, and Anti-Swarming Properties of *Hibiscus sabdariffa* L. Calyx Extracts: *In Vitro* and *In Silico* Modelling Approaches

**DOI:** 10.1155/2022/1252672

**Published:** 2022-05-20

**Authors:** Bechr Hamrita, Noumi Emira, Adele Papetti, Riadh Badraoui, Lamjed Bouslama, Mohamed-Iheb Ben Tekfa, Assia Hamdi, Mitesh Patel, Abdelbaset Mohamed Elasbali, Mohd Adnan, Syed Amir Ashraf, Mejdi Snoussi

**Affiliations:** ^1^Research Unit UR17ES30 “Virology & Antiviral Strategies”, Institute of Biotechnology, University of Monastir, Monastir, Tunisia; ^2^Department of Biology, College of Science, University of Hail, Hail, P.O. Box 2440, Saudi Arabia; ^3^Laboratory of Bioresources: Integrative Biology & Recovery, High Institute of Biotechnology, University of Monastir, Monastir, Tunisia; ^4^Laboratory of Nutraceutical & Food Chemical-Toxicological Analysis, Department of Drug Sciences, University of Pavia, Pavia, Italy; ^5^Section of Histology-Cytology, Medicine Faculty of Tunis, University of Tunis El Manar, Road Djebel Lakhdar, 1007 La Rabta, Tunis, Tunisia; ^6^Laboratory of Bioactive Substances, Center of Biotechnology of Borj Cedria, University of Tunis El Manar, Tunisia; ^7^Laboratory of Chemical, Pharmaceutical and Pharmacological Development of Drugs, Faculty of Pharmacy of Monastir, University of Monastir, Monastir, Tunisia; ^8^Department of Biotechnology, Parul Institute of Applied Sciences and Centre of Research for Development, Parul University, Vadodara 391760, Gujarat, India; ^9^Department of Clinical Laboratory Science, College of Applied Sciences-Qurayyat, Jouf University, Sakakah, Saudi Arabia; ^10^Department of Clinical Nutrition, College of Applied Medical Sciences, University of Hail, Hail, P.O. Box 2440, Saudi Arabia; ^11^Laboratory of Genetics, Biodiversity and Valorisation of Bioresources, High Institute of Biotechnology, University of Monastir, Monastir, Tunisia

## Abstract

The aim of this study was to investigate the phytochemical composition of dried Roselle calyx (*Hibiscus sabdariffa* L.) using both ethanolic and aqueous extracts. We report the antimicrobial activities against a wide range of bacteria, yeast, and fungi. The antioxidant activities were tested using 2,2-diphenyl-1-picrylhydrazyl (DPPH), hydroxyl, and 2–2′-azinobis-(3-ethylbenzthiazoline-6-sulfonic acid) radical scavenging assays. We report also for the first time the effect of the swarming motility in *Pseudomonas aeruginosa* PAO1. Our results showed that the tested two extracts were a rich source of phenols, flavonoids, and tannins with different degrees. Additionally, eleven phytoconstituents were identified by LC/MS technique (*Hibiscus* acid: 3-caffeoylquinic acid, 5-caffeoylquinic acid, 5-feruloylquinic acid, cyanidin 3-o-glucoside, myricetin, quercetin 7-o-rutinoside, quercetin 3-o-glucoside, delphinidin 3-o-sambubioside, and kaempferol 3-o-p-coumaroyl-glucoside). Also, it was shown that the calyx extract can scavenge 86% of the DPPH radical, while the rate of 53% and 23% of inhibition of the DPPH was obtained only at the concentration of 125 and 50 *µ*g/mL, and a small inhibition was made at a concentration of 5 *μ*g/mL. Roselle extracts inhibited the growth of the selected microorganisms at low concentrations, while higher concentrations are needed to completely kill them. However, no activity against CVB-3 was recorded for both extracts. In addition, the obtained extracts reduced the swarming motility of *P. aeruginosa* at 2.5 mg/ml. The docking simulation showed acceptable binding affinities (up to −9.6 kcal/mol) and interaction with key residues of 1JIJ, 2QZW, and 2UVO. The obtained results highlighted the potential use of Roselle extract as a source of phytoconstituents with promising antimicrobial, antioxidant, and anti-quorum sensing activities.

The article "Phytochemical Analysis, Antioxidant, Antimicrobial, and Anti-Swarming Properties of Hibiscus sabdariffa L. Calyx Extracts: In Vitro and In Silico Modelling Approaches" was published in 2022. Journal: Evid Based Complement Alternat Med.

## 1. Introduction

The plants still show a beneficial role in the treatment of various human pathologies. Isolation and extraction of plant compounds are imperative to understand their impact on the prevention and treatment of serious illness [1]. Several reports have been executed on natural antioxidants for decades to decipher protection against diseases linked to powerful oxidative stress and to the various damages induced by the presence of free radicals. Generally, oxidative stress is associated with several diseases, including cancer, neurodegenerative diseases, diabetes and inflammatory diseases, and aging process [2].

Actually, it has been proven that plants have shown a various range of compounds with antioxidant activities such as polyphenols as secondary metabolites. This component has been shown as strongly natural antioxidants of the vegetable world [3]. Currently, they are used against heart conditions, headaches, colds, wounds, and various skin infections, as well as insecticides and herbicides [4]. Natural phytocompounds can offer us a possible alternative to antibacterial agents [5].

In other way, previous studies have shown also that plants and their derived extracts are effective and may be of potential to inhibit bacterial QS system and biofilm [6]. In fact, QS and biofilm installation among resistant bacteria prove a major problem in human existence [7]. Several works have shown that resistance among bacteria or in QS and biofilm formation has motivated the treatment with plants and their derived extracts. Plants and their different extracts have been used to treat bacterial aggression and used as anti-QS compounds [6]. QS plays a crucial role in biofilm installation and virulence factor production [8].

The article "Phytochemical Analysis, Antioxidant, Antimicrobial, and Anti-Swarming Properties of Hibiscus sabdariffa L. Calyx Extracts: In Vitro and In Silico Modelling Approaches" was published in 2022. Journal: Evid Based Complement Alternat Med.

*Hibiscus sabdariffa L*. (HS) is a plant from the Malvaceae family, which normally grows in subtropical and tropical regions around the world. “*Zobo*” is a local drink known in Nigeria from a medicinal herb HS, used in folk medicine to treat hypertension [4]. Various works have been carried out targeting the physiological effects of its calyces, focused on various aqueous and organic extracts rich in bioactive compounds such as tocopherols, polyphenols, flavonoids, and organic acids such as malic acids, oxalic acids, and also shikimic acid [9].

Extracts from the HS calyces have shown several essential biological activities and may include antibacterial properties. *In vitro* studies have proven the effectiveness of HS in inhibiting pathogenic strains such as *E. coli*. The aqueous, ethanolic, and methanolic extracts from HS have shown good efficacy against enterohemorrhagic *E. coli* (EHEC) O157:H7 [10]. In addition, other researchers have noted that the methanolic extract from HS has potent bactericidal activity against clinical isolates of uropathogenic *E*. *coli* (UPEC) [11].

Another study revealed that the aqueous extract of HS shows an inhibitory effect against *Ascaris galliavium* in poultry. In addition, the coloring part from the calyces would also be fatal for *Mycobacterium tuberculosis* [12]. Roselle has also shown significant effects in India, such as aphrodisiac, astringent, cholagogue, demulcent, digestive, diuretic, emollient, purgative, refrigerant resolvent, sedative, stomachic, and tonic. Roselle is noted also as being a popular treatment for abscesses, bilious conditions, coughs, dysuria, scurvy, and cancer [11, 13–15]. According to the literature, several studies have proven its uses in the treatment of different diseases such as cancer, abscesses, bilious conditions, and cough, pathologies directly linked to microbial infections [16]. *In vivo* studies have shown that the anthocyanins of Hibiscus, a part of natural phenolic pigments present in the dried flower of Roselle and *H. rosa-sinensis*, have proven cardioprotective, hypocholesterolemic, and heapatoprotective effects [5].

In addition, other phenolic compounds, which have been isolated from dried HS flowers such as anthocyanin pigments and other phenolic compounds (*Hibiscus* protocatechuic acid), have shown that a protective role against tert-butyl hydroperoxide (t-BHP) induces oxidative stress, so hepatotoxicity has been noted *in vitro* and *in vivo* [17]. In addition, other work has shown that polyphenols, which are extracted from HS, have the ability to inhibit the accumulation and storage of triglycerides, to minimize the harmful effect of oxidative damage and the secretion of inflammatory adipokines, which directly target the infiltration of macrophages into adipose tissue [18, 19]. *In vitro*, the polyphenolic extract from HS has shown remarkable efficiency. These studies have shown that these compounds prevent fatty liver in hyperlipidemic mice by regulating gene expression applied in the regulation of glucose and lipid homeostasis and by lowering blood pressure and regulating endothelial function [18, 20].

The article "Phytochemical Analysis, Antioxidant, Antimicrobial, and Anti-Swarming Properties of Hibiscus sabdariffa L. Calyx Extracts: In Vitro and In Silico Modelling Approaches" was published in 2022. Journal: Evid Based Complement Alternat Med.

To find new therapeutic resources with a powerful antioxidant effect, the objective of this work was to assess the antioxidant potentials, the antimicrobial activities, and the anti-swarming properties of the aqueous methanolic compounds of *H. sabdariffa* in relationship with its phytochemical composition. Furthermore, the intermolecular interactions of *H. sabdariffa* identified compounds and some targeted receptors (1JIJ, 2QZW, and 2UVO) were assessed using *in silico* molecular docking approach.

## 2. Materials and Methods

### 2.1. Preparation of the Extracts

The fresh parts of the Roselle were collected in March 2017 in Biskra (Algeria). In the laboratory, the collected parts of Roselle calyces were washed with sterile distilled water. Ten grams of the powdered dried plant material was soaked in 100 ml of pure methanol or pure distilled water for 48 h. The homogenate was filtered using Whatman's filter paper. The final solution was concentrated, and the methanol was removed using a rotary evaporator. The small volume was later freeze-dried and kept in the freezer at 4°C for further studies.

### 2.2. Biological Material

In this work, the antifungal activity of the different extracts was tested against several fungi belonging to the genera *Aspergillus*, *Fusarium,* and *Penicillium* including the species *Aspergillus niger* DSM 63263, *Fusarium oxysporum*, *Penicillium expansum* DSM 994, *P. citrinum* DSM 1997, *P. simplicissimum* DSM 1097, *A. versicolor* DSM 1993, and *A. niger*. Four yeast strains were also tested namely *Candida albicans* ATCC 2019, *C. parapsilosis* ATCC 22019, *C. kefyr* ATCC 6258, and *C. tropicalis* ATCC 06–085. The antibacterial activity was tested against nine bacterial strains frequently isolated from human infections and food poisoning: *Staphylococcus aureus* ATCC 25923, *S. epidermidis* CIP 106510, *Escherichia coli* ATCC 35218, *Listeria monocytogenes* ATCC 19115, *Pseudomonas aeruginosa* ATCC 27853, *Enterococcus faecalis* ATCC 29212, *Salmonella typhimurium* ATCC 1408, *Bacillus cereus* ATCC 11778, and *Vibrio parahaemolyticus* ATCC 17802. For cytotoxicity and antiviral activities, Vero cells, herpes virus type 2, and Coxsackievirus type 3 were used.

The article "Phytochemical Analysis, Antioxidant, Antimicrobial, and Anti-Swarming Properties of Hibiscus sabdariffa L. Calyx Extracts: In Vitro and In Silico Modelling Approaches" was published in 2022. Journal: Evid Based Complement Alternat Med.

### 2.3. Phytochemical Screening of *H. sabdariffa* Extracts

#### 2.3.1. Polyphenol's Evaluation

The Folin-Ciocalteu protocol [21] was used for the evaluation of total phenolic compounds in selected parts of plants. For the experiment, 1000 *μ*L of extracts was added to 5 ml of Folin-Ciocalteu reagent (mixed with distilled water 1 : 10 v/v) and 4 ml (75 g/L) of sodium carbonate. The samples were vortexed for 15 s and left to stand for 30 min at 40°C for staining. The absorbance was determined at a wavelength of 765 nm using the Thermo Scientific Spectrascan UV 2700 dual-beam spectrophotometer. The concentration of each plant extract was 0.1 g/ml. Phenol levels were calculated in mg/g of n-propyl gallate equivalent.

### 2.4. Flavonoid Estimation

The level of total flavonoids was determined using the procedure already described by Haddaji et al. [21]. In summary, 2 mL of distilled water and a NaNO_2_ (0.15 ml; 5%) solution were added to 0.5 ml of plant extract. After 6 min of incubation at room temperature, a solution of AlCl_3_ (0.15 ml, 1.1%) was added and allowed to stand for six minutes. Subsequently, a solution of NaOH (2 ml, 4%) was added to the mixture. Immediately, the distilled water was added (5 ml). Then, the mixture is allowed to stand for 15 minutes, and the color intensity was measured at 510 nm. The results were reported in mg of catechin equivalent (EC) per gram of the extract.

### 2.5. Determination of Total Tannins

The quantification of total tannins in both extracts was estimated using the same protocol described by Haddaji et al. [21]. For the experiment, 50 *μ*l of each extract was appropriately diluted and mixed with a volume of 1.5 ml of 4% vanillin and then added to 750 *μ*l of concentrated HCl. After vigorous stirring, the mixture was incubated for 20 min at room temperature. Then, the absorbance was measured at 500 nm [22]. The contents of condensed tannins are expressed in mg of equivalent catechin per gram of extract.

### 2.6. RP-HPLC-DAD-ESI-MS^n^ Analysis

To obtain a profile of polyphenolic composition of methanolic and aqueous extracts, an HPLC-DAD-ESI/MS^n^ analysis was carried out. Ten milligrams of dried samples was solubilized in 10 ml of the mobile phase, and 5 *µ*l was injected in the Thermo Finnigan Surveyor Plus HPLC System (Thermo Fisher Scientific, Waltham, MA), equipped with a Surveyor UV-Vis photodiode array detector (PAD), connected to an LCQ Advantage MAX ion trap mass spectrometer through an ESI source (Thermo Fisher Scientific, Waltham, MA). The analysis was performed on a Gemini C18 analytical column (150 mm × 2.0 mm i.d., 5 *μ*m) with a Hypersil GOLD C18 guard column (10 mm × 2.1 mm i.d., 5 *μ*m; both from Phenomenex, Torrance, CA). A binary mobile phase was used, and it consisted of eluents A and B, which were 0.1% formic acid aqueous solution and acetonitrile, respectively. Analytes were eluted in a linear gradient from 5% to 95% B in 70 min at a flow rate of 0.3 ml/min, 30°C. Each run was followed by column reconditioning. The chromatogram was recorded at 315 nm (hydroxycinnamic acids), 370 nm (flavonols), and 520 (anthocyanins). Spectral data were acquired in the range of 190–600 nm for all peaks. The ion trap was operated in data-dependent, full-scan (100–1800 *m/z*), and MS/MS mode to obtain fragment ions (*m/z*) with a collision energy of 30% and an isolation width of 3 *m/z*. ESI source parameters were optimized to an ionization voltage of 4 kV, a capillary temperature of 320°C, a sheath gas flow rate of 15 arbitrary units, and an auxiliary gas flow rate of 10 arbitrary units. Thermo Fisher Scientific Excalibur 2.0 software was used for data acquisition and processing.

The article "Phytochemical Analysis, Antioxidant, Antimicrobial, and Anti-Swarming Properties of Hibiscus sabdariffa L. Calyx Extracts: In Vitro and In Silico Modelling Approaches" was published in 2022. Journal: Evid Based Complement Alternat Med.

### 2.7. Antioxidant Activities of *H. sabdariffa* Extracts

The antioxidant activity of the extracts was studied by three methods: the trapping power of the free radical DPPH, that of the radical ABTS, and the power of reduction of ferric ions (FRAP).

### 2.8. Scavenging Activity of DPPH Radical

The DPPH radical scavenging activity was evaluated using the protocol of Moraes-de–Souza et al. [23] after rectifications. The reaction was composed of 30 *μ*l of extract, 3 ml of methanol, and 0.270 ml of a solution of 0.5 mM 2,2-diphenyl-1-picrylhydrazyl (DPPH) radical solution in methanol. The absorbance was measured in an ELx800 microplate reader (BioTek Instrument, Inc., Winooski, VT, USA) at 517 nm, after 45 min of incubation. The antioxidant activity was calculated using the following equation:

(1) $$\begin{array}{c} \%\text{inhibition}=\left[\frac{\left(A\text{ control}-A\text{ sample}\right)}{A\text{ control}}\right]\times 100, \end{array}$$

where *A*_control_ = absorbance of negative control at the moment of solution preparation and *A*_sample_ = absorbance of sample after 45 min.

The antioxidant activity was expressed as IC_50_ (mg/mL), which represented the extract concentrations scavenging 50% of DPPH radicals [21].

### 2.9. Scavenging Activity of ABTS Radical

The ABTS radical scavenging activity was evaluated using the protocol referred to Re et al. [24] after rectifications. 7 mM of 2,2′-azinobis (3-ethylbenzothiazoline-6-sulfonic acid) (ABTS) was added to the distilled water. The radical cation ABTS (ABTS ∙ +) was generated in the presence of ABTS and 2.45 mM potassium persulfate (final concentration), and then, the mixture will be placed in the dark at room temperature for 12 to 16 h before use.

The article "Phytochemical Analysis, Antioxidant, Antimicrobial, and Anti-Swarming Properties of Hibiscus sabdariffa L. Calyx Extracts: In Vitro and In Silico Modelling Approaches" was published in 2022. Journal: Evid Based Complement Alternat Med.

The dilution of the ABTS^+^ solution was performed with water to an absorbance of 0.70 (±0.02) at 734 nm. The reaction mixture is composed of 0.07 ml of the HS extract and 3 ml of the ABTS radical. Then, this mixture is incubated for 7 min, and the absorbance reading was taken using a spectrophotometer at 734 nm. The antioxidant activity was calculated using the following equation:

(2) $$\begin{array}{c} \%\text{inhibition}=\left[\frac{\left(A\text{ control}-A\text{ sample}\right)}{A\text{ control}}\right]\times 100, \end{array}$$

where *A*_control_ = absorbance of negative control at the moment of solution preparation and *A*_sample_ = absorbance of sample after 6 min.

The EC_50_ values were evaluated from the curves, which show the concentration of the extract required to scavenge 50% of the free radical ABTS. The EC_50_ is generally defined to determine the amount or concentration of extracts required to scavenge 50% of free radicals.

### 2.10. Ferric Reducing Antioxidant Power (FRAP) Methods

This technique is based on the microplate reader. Indeed, volumes of the order of 0.5 ml of the different concentrations of the extracts tested were mixed with a sodium phosphate buffer (200 mmol/l, pH 6.6, 0.5 ml) and ferricyanide of potassium (1% *w*/*v*, 0.5 ml). The mixture was incubated at 50°C for 20 minutes, and then, trichloroacetic acid (10% *w*/*v*, 0.5 ml) was added. Afterwards, 0.8 ml of the mixture was poured into the 48-well microplates, and then, the deionized water (0.8 ml) and the ferric chloride (0.1% *w*/*v*, 0.16 ml) were added. Absorbance was measured at 690 nm. The concentration of the extract, which gives 0.5 absorbance (EC_50_), was estimated from the graph, which reports the evaluation of the absorbance at 690 nm as a function of the concentrations of the extract.

### 2.11. Screening for Antimicrobial Activities

#### 2.11.1. Disc Diffusion Method

Antibacterial activity was carried out by the disc diffusion method [25] against nine Gram-positive and Gram-negative type bacterial strains. The same technique was used to study the antifungal activity of HS extracts against four *Candida* species on Sabouraud chloramphenicol agar plate at 30°C for 17–26 h.

The optical density of all bacteria was adjusted to 0.5 McFarland turbidity standards and 2 McFarland for yeast strains with a DENSIMAT (bioMérieux). The suspension was used to inoculate Mueller Hinton/Sabouraud chloramphenicol Petri dishes using a sterile cotton swab. The plant extract was prepared at a final concentration of about 100 mg/ml. Sterile filter paper discs (6 mm in diameter) were impregnated with 10 *µ*l of plant extract that was placed on the cultured plates. After 1.5–3 h at 4°C, the treated Petri dishes were incubated at 27 or 36°C for 17–24 h. For fungi, a spore solution (10^6^ spore/mL) was used to inoculate the potato dextrose agar Petri dishes that were incubated for 48 h at 37°C.

The article "Phytochemical Analysis, Antioxidant, Antimicrobial, and Anti-Swarming Properties of Hibiscus sabdariffa L. Calyx Extracts: In Vitro and In Silico Modelling Approaches" was published in 2022. Journal: Evid Based Complement Alternat Med.

The treated Petri dishes were placed at 4°C for 1.5–3 h and then incubated at 37°C for 17–24 h. The inhibition of microorganism growth was evaluated by measuring the diameter of the transparent inhibition zone around each disc. The average of three measurements was recorded. The susceptibility of the standard (ampicillin and amphotericin B) was determined at a final concentration of about 10 mg/disc.

### 2.12. Microdilution Assay

The determination of MICs and MBCs was performed by dilution technique in a liquid medium used for bacteria [25], yeast [26], and fungi [27]. For the experiment, 95 *μ*l of Sabouraud broth (yeast and fungi) or Mueller Hinton broth (bacteria), 5 *μ*l of bacterial or fungal suspension, and 100 *μ*l of dilution of the extract were tested. The negative control well contains 195 *μ*l of enrichment broth without extract and 5 *μ*l of suspension of the microorganism to be tested. The final volume in each well is 200 *μ*l. After incubation at 37°C for 24 h for bacteria and yeast and 48 h for fungi, the lowest concentration, at which there was no turbidity, was also regarded as MIC value of the extract. MBC/MFC is defined as the concentration of extract that totally inhibits the growth of microorganisms tested confirmed on MH/SC/PDA agar. According to Zahin et al. [28], plant extract exerted two types of activities: a bacteriostatic/fungistatic (MBC/MIC ≥4) and bactericidal/fungicidal activity (MBC/MIC <4).

### 2.13. Study of Antiviral Activity

Vero cells (ATCC No. CCL-81) were cultivated in RPMI 1640 supplemented with 10% fetal bovine serum (FBS) mixed with 1% penicillin (100 U/ml), 1% streptomycin (100 mg/ml), and 1% fungizone (2.5 mg/ml). Vero cells were grown in a solution composed of RPMI containing 5% FBS, placed in sterile 96-well, 24-well flat-bottomed plates at 1 g/10^4^ cells/well, at 37°C, and incubated under 5% CO_2_ humidified atmosphere at 37°C.

The stock solutions were diluted serially with RPMI media without FBS to obtain many extract concentrations. In general, the final concentration of DMSO in the working concentration was below 0.5%. The determination of the cytotoxic concentration of the two extracts was performed on 96-well flat-bottomed plates. One hundred *µ*l of ½ diluted extracts starting from 2.5 mg/mL concentration was deposited on cells in confluence. Vero cells treated with 0.5% DMSO in PBS were used as negative control. All experiments were performed in triplicates. Then, the plate was incubated under 5% CO_2_, humidified atmosphere at 37°C. After 72 h, the extract dilutions were substituted with 100 *µ*L of the MTT solution (5 mg/mL) and incubated for 4 h at 37°C. Then, the formazan crystals were dissolved with DMSO and the plate was read on an ELISA reader at a 570 nm wavelength to measure the optical density. 50% cytotoxic concentration (CC_50_) of crude plant extracts, which is the concentration that causes 50% cell cytotoxicity of Vero cells, was determined by linear regression.

The article "Phytochemical Analysis, Antioxidant, Antimicrobial, and Anti-Swarming Properties of Hibiscus sabdariffa L. Calyx Extracts: In Vitro and In Silico Modelling Approaches" was published in 2022. Journal: Evid Based Complement Alternat Med.

### 2.14. Viruses and Antiviral Activity

Antiviral activity was performed on the same 96-well flat-bottom plates. Confluent Vero cells were infected with 50 TCID_50_ (50% tissue culture infective dose) of CVB-4 in the presence of 100 *µ*l of ½ diluted extracts starting from CC_50_. Following 1 h of incubation, the medium was removed, and the cells were washed with PBS. Vero cells infected without extract were used as a virus control. All experiments were performed in triplicates. Then, the plate was incubated under 5% CO_2_ humidified atmosphere at 37°C. After 48 h, the medium was substituted with 100 *µ*L of the MTT solution (5 mg/mL) and incubated for 4 h at 37°C. Then, the formazan crystals were dissolved with DMSO and the plate was read on an ELISA reader at a 570 nm wavelength to measure the optical density. 50% inhibitory concentration (IC_50_) of crude plant extract, which is the concentration that reduces the optical density by 50% in comparison with the cell control, was determined by linear regression.

### 2.15. Anti-Swarming Motility Test

In swarming assays, overnight cultures of the test bacteria (*P. aeruginosa* ATCC 27853) were point inoculated (5 *μ*l) at the center of swarming plates consisting of 1% peptone, 0.5% NaCl, 0.5% agar, and 0.5% of filter-sterilized D-glucose with various concentrations of Hibiscus aqueous methanolic extracts (0.5, 1, 2.5, and 10 mg/ml). The plate without the extract was maintained as control. The plates were incubated at an appropriate temperature in the upright position at 37°C for 18 h. The swarming migration was recorded by following swarm fronts of the bacterial cells.

### 2.16. In Silico Molecular Docking and Intermolecular Interactions

The biological activity of the compounds identified by RP-HPLC-DAD-ESI-MS^n^ analysis was confirmed by *in silico* molecular docking and interaction assay. The active sites of some selected receptors (TyrRS from *S. aureus*; PDB ID : 1JIJ, aspartic proteinase from Candida albicans, PDB ID : 2QZW, and wheat germ agglutinin, PDB ID : 2UVO) have been targeted to assess the antibacterial/antimicrobial and antiviral effects, respectively. The tridimensional structures of the targeted proteins were obtained from RCSB. ChemDraw was used to draw the chemical structures of the previously identified 17 compounds [29, 30]. The docking approach was based on the CHARMM force field after processing ligands and receptors: polar hydrogen and Kollman charges. The binding affinity and the hydrogen bond calculations were assessed as previously reported [29, 31–33]. These receptors have been selected because they are highly involved in the bacterial, viral, and quorum sensing processes and are commonly targeted in pharmaceutical studies as they are parts of the treatment pathways [34, 35].

The article "Phytochemical Analysis, Antioxidant, Antimicrobial, and Anti-Swarming Properties of Hibiscus sabdariffa L. Calyx Extracts: In Vitro and In Silico Modelling Approaches" was published in 2022. Journal: Evid Based Complement Alternat Med.

### 2.17. Statistical Analysis

All the analyses were run in triplicate and averaged. All values are expressed as mean ± standard deviation. The CC_50_, EC_50_, and IC_50_ values were estimated by extrapolating the graph plotted with software Microsoft Excel 2007. Mean values were compared using multiple comparison of Duncan's test with the SPSS statistical software program (SPSS v.16). The difference was statistically significant when *p* < 0.05.

## 3. Results

### 3.1. Phytochemical Composition of the Obtained Extracts

The phytochemical composition of both methanolic and aqueous extracts of Hibiscus calyces is summarized in Table 1. Phenolic compounds are secondary metabolites whose presence is highly influenced by environmental and genetic factors. Their contents vary according to the plant and/or studied organ. Indeed, the methanolic extract of Hibiscus has a polyphenol content in the order of 19.58 ± 0.08 mg EAG/g of dry extract, which has been found to be lower than the aqueous extract of the same plant of 22.71 ± 0.08 mg EAG/g of dry extract.

According to the results obtained, it is noted that the flavonoids are the most abundant phenolic compounds in the flower of Hibiscus with an amount of 22.49 ± 1.04 mg EC/g of the aqueous extract. The extracts showed also low content of tannin molecules. These values are in the order of 8.4 ± 0.7 mg EC/g of the dry extract for the aqueous extract and about 1.16 ± 0.16 mg EC/g of dry extract for the methanolic extract of the Hibiscus calyces.

A list of compounds identified in methanolic and aqueous extracts by LC-MS is reported in Table 2. The methanolic extract contained two anthocyanins, which were detected in positive ionization mode, i.e., delphinidin 3-*O*-sambubioside (compound 10) and cyanidin 3-*O*-glucoside (compound 6). Both of them fragmented giving the aglycone ions at *m/z* of 303 and 287, which corresponded to the loss of sambubiose and glucose moieties, respectively. Four flavonols were also detected. Myricetin (compound 7) ionized to give an ion at *m/z* of 319, and it was confirmed by comparing its behavior with that of the standard, as well as the identity of quercetin 3-*O*-glucoside (*m/z* 465) (compound 9). Another quercetin derivative (compound 8) was present; it fragmented giving a base peak an ion at *m/z* of 303 and a very intense parent ion at *m/z* of 302, thus indicating the linkage position of the sugar moiety on the aglycone and leading to the correct identification of the disaccharide [39]. Kaempferol 3-O-*p*-coumaroyl-gucoside (compound 11) was identified thanks to its fragmentation pattern, which was consistent with the loss of the glucose and of the acyl-glucose moieties, respectively.

The article "Phytochemical Analysis, Antioxidant, Antimicrobial, and Anti-Swarming Properties of Hibiscus sabdariffa L. Calyx Extracts: In Vitro and In Silico Modelling Approaches" was published in 2022. Journal: Evid Based Complement Alternat Med.

### 3.2. Biological Activities of the Different Extracts Obtained

#### 3.2.1. Antimicrobial Activity

The antimicrobial activities were evaluated using the disc diffusion test to determine the diameters of the bacterial growth inhibition zones. The liquid microdilution assay was carried out to evaluate the minimum inhibitory concentrations (MICs) and the minimum bactericidal concentrations (MBCs). The inhibition of microbial growth (bacteria and yeasts) resulted in the appearance of a halo around each disc impregnated with the extract to be tested.

The results of the agar diffusion assay reveal that the antibacterial activity of the extracts is dependent from the target bacterium. Indeed, the Hibiscus aqueous extract showed moderate antimicrobial activity with a diameter zone inhibition of 18.33 mm. It is noted that the highest antimicrobial activity was obtained with the same extract against *L*. *monocytogenes* strain ATCC 19115 with a mean zone of growth inhibition value of 21 mm. In fact, the Hibiscus methanolic extracts showed a zone inhibition of 17.12 mm. According to studies confirmed by Kalemba and Cunicka [41], the sensitivity of a microorganism certainly depends on the composition variability of the extract and also of the microorganism itself. The antifungal activity has shown variation in growth inhibition. In fact, the inhibition diameter of yeast with methanolic extract was about 14 mm; however, it was ranging from 14 to 17 mm, when the aqueous extract was used. All these results are summarized in Table 3.

The determination of MICs and MBCs/MFCs showed that the Hibiscus extracts in liquid medium are very active on all tested bacteria and yeasts but with different degrees. In addition, these extracts appear to be more effective on bacteria than yeasts with lower MICs and MBCs compared with those recorded for yeasts. In the liquid medium, the lowest MIC values are recorded with the Hibiscus aqueous extract (MICs: 9.375 mg/ml) and the lowest CMFs by the same plant methanolic extract (MFCs: 18.75 to 37.5 mg/ml). It is the same for the bacteria tested by the Hibiscus aqueous extract with similar MICs in all bacteria (2,342 mg/ml) and CMBs ranging from 4.68 to 9.375 mg/ml. All these results are expressed in Table 3. The antifungal activity results of the different methanolic and aqueous extracts tested on two strains of fungi according to the microdilution method recorded that the minimum inhibitory concentrations vary from 75 to 150 mg/ml (Table 4).

The article "Phytochemical Analysis, Antioxidant, Antimicrobial, and Anti-Swarming Properties of Hibiscus sabdariffa L. Calyx Extracts: In Vitro and In Silico Modelling Approaches" was published in 2022. Journal: Evid Based Complement Alternat Med.

### 3.3. Cytotoxicity and Antiviral Activities

*Hibiscus* extracts showed low cytotoxicity on Vero cell lines with CC_50_ of 946 and 1250 *μ*g/ml, respectively, for methanolic and aqueous extracts. However, no activity against CVB-3 was recorded for both extracts.

### 3.4. Study of the Antioxidant Activity of the Extracts Obtained

The antioxidant activity of the extracts was evaluated by the DPPH method. This method makes to evaluate the ability of phenolic compounds to inhibit the DPPH radical. The results showed that both Roselle extracts were able to scavenge the DPPH free radical with different degrees (IC_50_ value about 2.793 ± 0.044 mg/ml for methanolic extract and 2.471 ± 0.024 mg/ml for the aqueous one). For the radical ABTS+^*∗∗*^, the results obtained showed that the Hibiscus methanolic extract has the highest antioxidant activity with an EC_50_ value of 1.918 ± 0.06 mg/ml as compared to its aqueous extract of 2.082 ± 0.0035 mg/ml. The presence of reducing agents in plant extracts causes the Fe^3+^/ferricyanide complex to be reduced to the ferrous form. The results obtained show that the Hibiscus aqueous and methanolic extracts have low EC_50_ values of about 0.578 ± 0.016 and 0.676 ± 0.026 mg/ml, respectively. All these data are summarized in Table 5.

### 3.5. Anti-Quorum Sensing Activity

#### 3.5.1. Anti-Swarming Activity

Swarming migrations play an important role in quorum sensing biofilm formation, and we tried to examine the anti-QS potential of Hibiscus aqueous and methanolic extracts against motility in PAO1 strain. Our results indicated that HS extracts inhibited the swarming of PAO1 at the three tested concentrations (2.5, 5, and 10 mg/ml) (Figure 1). However, a high inhibition in the migration of PAO1 was obtained at 2.5 mg/ml. At high concentration of both tested extracts, a reduction in the intensity of the green coloration of the pigment “pyocyanin” was noted. All these data are summarized in Table 6.

### 3.6. In Silico Results

The molecular interactions of the plant-identified compounds and some targeted macromolecules involved in the biological activities are reported in Table 7. The in silico data reported in this study correspond to the better positions with both best binding affinity and RMSD equal to zero, as commonly reported in molecular interactions' studies [42–44]. The compounds were predicted to establish different biding affinities reaching −9.6 for 1JIJ, −7.5 for 2QZW, and −6.9 for 2UVO. This might be related to the structure-activity relationship [30, 32, 33, 43]. Figures 2–4 exhibit 3D and 2D illustrations of the top 3 complexes with the highest binding scores.

The article "Phytochemical Analysis, Antioxidant, Antimicrobial, and Anti-Swarming Properties of Hibiscus sabdariffa L. Calyx Extracts: In Vitro and In Silico Modelling Approaches" was published in 2022. Journal: Evid Based Complement Alternat Med.

## 4. Discussion

Hydroxycinnamic acid derivatives were the compounds mostly present in the aqueous extract in addition to a less concentration of compounds 7, 8, 9, and 11. In fact, two different isomers of caffeoylquinic acids (CQAs) were detected and they were identified as 3-CQA (compound 3) and 5-CQA (compound 4) according to the different intensities of a fragment ion at *m/z* of 179 and the presence of an ion at *m/z* of 135 only in MS/MS fragmentation of 3-CQA [45]. A similar fragmentation pattern was registered for compound 5, identified as 5-feruloylquinic acid. Another caffeic acid derivative was present and its fragmentation gave as the base peak an ion at *m/z* of 179, indicating a hexose linked to the acidic moiety (compound 2). Hibiscus acid (compound 1) was also present; it is the lactone derivative of hydroxycitric acid and fragment losing a water molecule and the CO_2_. The presence of these molecules in *Hibiscus* extracts was already reported in the literature with the exception of cyanidin 3-*O*-glucoside; in fact, the sambubioside derivative was generally detected [36, 46, 47].

The obtained results are in agreement with those previously described in the international bibliography concerning these two studied plants. In this way, it has been demonstrated that the crude extract of *Hibiscus* plant has an antibacterial activity directed against strains of *Streptococcus mutans* isolated from the oral cavity with a minimal inhibitory concentration in the order of 2.5 mg/ml [48] and the species of *Campylobacter* sp. (*Campylobacter jejuni, Campylobacter coli, and Campylobacter fetus*) that contaminate beef, pork, and poultry meat with inhibitory concentrations ranging from 96 to 152 *μ*g/ml [49]. In addition, Olaleye and Rocha [50] have shown that the methanol Hibiscus water extract has antibacterial activity against several Gram-positive and Gram-negative bacteria including the following species: *S. aureus, Bacillus stearothermophilus, Micrococcus luteus, Serratia marcescens, Clostridium sporogenes, Escherichia coli, K. pneumoniae, Bacillus cereus, and P. fluorescence.* This author has also shown that this same extract is not active against yeast *Candida albicans* [50].

The article "Phytochemical Analysis, Antioxidant, Antimicrobial, and Anti-Swarming Properties of Hibiscus sabdariffa L. Calyx Extracts: In Vitro and In Silico Modelling Approaches" was published in 2022. Journal: Evid Based Complement Alternat Med.

In 2017, Quing et al. showed that the raw Hibiscus seed extract is active against three Gram-negative strains such as *Salmonella, Shigella,* and *Enterobacter*. In 2015, Borrás-Linares and his collaborators showed that the ethanolic extract of 25 varieties of Hibiscus was active against *E. coli, S. enteritidis*, *M. luteus,* and *S. aureus* strains with inhibition zones ranging from 16 to 22 mm for *S. aureus* and from 10 to 18 mm for *the M. luteus* strain. Gram-negative strains were the most resistant with an inhibition diameter ranging from 10 to 16 mm for both *E. coli* and *S. enteritidis* strains [10]. Recently, Abdallah [5] has shown that the Hibiscus methanolic extract of calyx grown in Sudan is active against antibiotic-resistant strains of *Acinetobacter baumannii* with inhibition zone diameters of 11.3 ± 0.3 and 13.6 ± 0.3 mm and MIC and MBC values ranging from 25 to 50 mg/ml and 50 to 100 mg/ml, respectively. *Hibiscus* extract has also been shown to have activity against strains of *C. albicans* isolated from urinary tract infections and to inhibit biofilm formation by this yeast [11].

Both extracts show a proportional increase in the inhibition percent of the DPPH radical depending on the used concentration. These inhibition percentages exceed 50% at very low concentrations of tested extracts. The inhibition percentages reveal a proportional decrease in the DPPH radical until its total disappearance at a concentration of 10 mg/ml for all the tested extracts. From the curves of the various extracts, the concentration of antioxidant necessary to remove 50% of a quantity of DPPH (at equilibrium), it is the effective concentration (EC_50_). The low EC_50_ values indicate the effectiveness of the extract and thus are a better and powerful antioxidant. The EC_50_ values calculated for the DPPH activity are 2.793 and 2.471 mg/ml for aqueous and methanolic HS extracts, respectively. The antioxidant activity is associated with the phenolic composition, which is in agreement with our results, since the extracts, which have higher phenolic compound contents, are the extracts having the more pronounced antioxidant activity [51]. The results recorded for the estimation of the anti-swarming activity proved that the tested extracts significantly decreased the mobility of PAO1.

The molecular docking approach showed that for H-bond interactions, which are considerably associated with pharmaceutical effects and drug design [29, 31, 32, 44], the highest number of H-bonds was found with Hibiscus acid (Lys^84^, Arg^88^, Arg^88^, Tyr^170^, Gln^174^, Gln^196^, Asp^80^, Gly^38^, Gln^196^, Asp^80^, and Gln^196^) and quercetin 3-O-glucoside (Asp^40^, Asn^124^, Gln^174^, Gln^174^, Gly^193^, Gln^196^, Asp^177^, Asp^177^, Asp^195^, Gly^49^, and Gln^190^). The latter complex was reinforced with a supplementary network of interactions involving His^50^ and Ala^39^ (twice for each) and Gly^38^ and Asp^40^ (once for each). These compounds established 11 conventional H-bonds with 1JIJ, particularly with some key residues such as Asp^40^, Asp^80^, and Gln^196^. Furthermore, all the compounds were deeply embedded within the pocket region and showed close vicinity to the targeted proteins. For instance, the close vicinity was predicted for 1JIJ-quercetin 7-O-rutinoside (1.57 Å), 2QZW-quercetin 7-O-rutinoside (1.47 Å), and 2UVO-3-caffeoylquinic acid (1.72 Å). In this context, it has been reported that closely related ligand-amino acid/receptor complexes may enhance the biological activity [31–33, 44]. Besides, for each targeted receptor, most of the identified compounds were predicted to occupy almost the same region, which may support the possible synergistic effects. In fact, it was reported that the use of the whole plant extract was suggested to be much better [32, 34, 43]. Overall, the in silico showed that the biological effect of *H. sabdariffa* compounds are thermodynamically possible. The computationally proved effects include (i) antibacterial via tyrosyl-tRNA synthetase from *S. aureus*, which is largely responsible for hospital-acquired infections [52]; (ii) antifungal as assessed against the secreted aspartic protease (SAP-1) of *C. albicans;* and (iii) antiquorum sensing through the wheat germ agglutinin. Such effects, explored using *in vitro* and/or *in vivo* approaches, would be of crucial importance and support our findings. The *in silico* findings, particularly the molecular interactions between ligands and receptors, would be confirmed and validated by molecular dynamic simulations.

The article "Phytochemical Analysis, Antioxidant, Antimicrobial, and Anti-Swarming Properties of Hibiscus sabdariffa L. Calyx Extracts: In Vitro and In Silico Modelling Approaches" was published in 2022. Journal: Evid Based Complement Alternat Med.

This study demonstrated also that both Hibiscus extracts inhibit the swarming motility of *P. aeruginosa* PAO1. Swarming motility is strongly involved in pathogenesis by aiding in the attachment of *P. aeruginosa* to the host tissue and colonizing the surfaces of the medical devices such as catheters [53]. Swimming is another major form of *P. aeruginosa* PAO1 motility, in which bacteria swim in aqueous environments via the flagellum [54]. *P. aeruginosa* exhibits swarming motility, which helps in initial attachment and later in relocation of biofilm from one site to another [55]. Moreover, swarming motility is important in early stages of biofilm formation by *P. aeruginosa* cells and confers to bacteria an extra advantage in tolerating the antibiotics [56]. In this study, it has been found that the exposure of PAO1 with Hibiscus extracts significantly impaired swarming motility of this bacterium. This finding is consistent with other studies that proved the repression of swarming of *P. aeruginosa* PAO1 by clove extracts and ginseng [57].

## 5. Conclusions

The results obtained indicate that *H. sabdariffa* L. is rich in natural antioxidant compounds, antimicrobial agent, and anti-swarming factor. Taken together, these biological properties may allow the tested extracts from *H. sabdariffa* to be considered as having the potential to be candidate in the design of new therapeutic strategies for microbial infections, and may lead to the development of novel bioactive molecules for industrial needs. Further studies, such as the use of other isolation and purification techniques of the active compounds and in *vivo* studies, would help to elucidate the mode of action of the observed beneficial effects of the aqueous and methanolic extracts.

## Figures and Tables

**Figure 1:** Anti-swarming activity of the methanolic and aqueous extracts from *H. sabdariffa* calyces tested against *P. aeruginosa* PAO1 strain. (a): methanolic extract and (b): aqueous extract; S: standard.

**Figure 2:** 3D illustration (a–c) and the corresponding 2D diagram of interactions (a'–c') for the compounds with the best docking scores of 13, 17, and 9 (−9.6, −9.4, and −9.1 kcal/mol) with the active site of 1JIJ.

**Figure 3:** 3D illustration (a–c) and the corresponding 2D diagram of interactions (a'–c') for the compounds with the best docking scores of 13, 17, and 9 (−7.8, −7.5, and −6.2 kcal/mol) with the active site of 2QZW.

**Figure 4:** 3D illustration (a–c) and the corresponding 2D diagram of interactions (a'–c') for the compounds with the best docking scores of 13, 8, and 11 (−6.9, −5.1, and −4.8 kcal/mol) with the active site of 2UVO.

**Table 1:** Phytochemical study of the methanolic and aqueous extracts from *H. sabdariffa* calyces. mg EGA/g extract: mg equivalent gallic acid/g extract; mg EC/g extract: mg equivalent catechin/g extract.

Compound	Aqueous extract (HE)	Methanolic extract (HM)
Total polyphenols (mg EGA/g extract)	22.71 ± 0.08	19.58 ± 0.08
Flavonoids (mg EC/g extract)	22.49 ± 1.04	16.3 ± 1.85
Tannins (mg EC/g extract)	8.4 ± 0.7	1.16 ± 0.10

**Table 2:** MS and MS/MS data of compounds detected in methanolic and aqueous extracts.

N	RT (min)	Precursor ion (*m/z*)	HPLC-ESI–MS^n^*m/z* (% of base peak)	Compound identity	References
**1**	12.90	189	MS^2^ [189]: 171 (20), 127 (100)	Hibiscus acid	Amaya-Cruz *et al.*, [36]; Rodriguez- Medina et al., [37]
**2**	34.21	341	MS^2^ [341]: 179 (100), 135 (20)	Caffeic acid derivative	Amaya-Cruz *et al.* [36]
**3**	37.62	353	MS2 [353]: 191 (100), 179 (60), 135 (10)	3-Caffeoylquinic acid	Carazzone *et al.*, [38]
**4**	38.22	353	MS2 [353]: 191 (100), 179 (10)	5-Caffeoylquinic acid	Carazzone *et al.*, [38]
**5**	39.92	367	MS2 [367]: 191 (100), 173 (25)	5-Feruloylquinic acid	Carazzone *et al.*, [38]
**6** ^**a**^	45.41	449^+^	MS^2^ [449]: 287 (100)	Cyanidin 3-O-glucoside	Amaya-Cruz *et al.*, [36]
**7** ^**a**^	54.50	319	—	Myricetin	Borrás-Linares *et al.*, [10]
**8**	62.47	611^+^	MS^2^ [611]: 303 (100), 302 (70), (100)	Quercetin 7-O-rutinoside	Shi *et al.*, [39]
**9** ^**a**^	65.02	465^+^	MS^2^ [465]: 303 (85), 303 (100)	Quercetin 3-O-glucoside	Rodriguez- Medina *et al.*, [37]
**10**	67.31	597^+^	MS^2^ [597]: 303 (100)	Delphinidin 3-O-sambubioside	Borrás-Linares *et al.*, [10]
**11**	72.56	595^+^	MS^2^ [595]: 449 (55), 287 (80), 286 (100)	Kaempferol 3-O-p-coumaroyl-glucoside	Fernández-Arroyo *et al.*, [40]

RT: retention time; ^a^compared with standard compound; ^+^positive ionization mode.

The article "Phytochemical Analysis, Antioxidant, Antimicrobial, and Anti-Swarming Properties of Hibiscus sabdariffa L. Calyx Extracts: In Vitro and In Silico Modelling Approaches" was published in 2022. Journal: Evid Based Complement Alternat Med.

**Table 3:** Determination of MICs, MBCs, and MBC/MIC ratio of *H. sabdariffa* methanolic and aqueous extracts compared with amphotericin and ampicillin.

	*H. sabdariffa* aqueous extract				*H. sabdariffa* methanolic extract				Ampicillin		
	IZ^*∗*^	MIC^*∗*^	MBC^*∗∗*^	MBC/MIC ratio	IZ	MIC	MBC	MBC/MIC ratio	IZ	MIC	MBC
*S. aureus* ATCC 25923	18 ± 0^*a*^	2.342	9.375	4	17 ± 1^*a*^	2.342	4.68	2	26.66 ± 1.15 ^*b*^	0.25	0.40
*S. epidermidis* CIP 106510	19 ± 2^*b*^	2.342	9.375	4	15.33 ± 0.57^*a*^	2.342	4.68	2	22.67 ± 0.57^*c*^	0.25	0.40
*E. coli* ATCC 35218	17 ± 1^*b*^	2.342	9.375	4	15 ± 1^*b*^	2.342	9.375	4	11.67 ± 1.52^*a*^	0.023	3
*L. monocytogenes* ATCC 19115	21 ± 1^*c*^	9.375	18.75	2	16.66 ± 0.57^*b*^	2.342	9.375	4	12.33 ± 0.57^*a*^	0.023	0.093
*E. faecalis* ATCC 29212	19.33 ± 0.57^*c*^	9.375	37.5	4	18 ± 0^*b*^	2.342	9.375	4	13.66 ± 0.57^*a*^	0.023	0.093
*S. typhimurium* ATCC 1408	18 ± 0^*a*^	9.375	>75	>4	17 ± 2^*a*^	2.342	9.375	4	17.33 ± 1.15^*a*^	0.023	0.093
*B. cereus* ATCC 11778	20 ± 2^*a*^	9.375	18.75	2	19.33 ± 0.57^*a*^	2.342	9.375	4	26.33 ± 1.52^*b*^	0.25	0.40
*V. parahaemolyticus* ATCC 17802	17.33 ± 0.57^*b*^	9.375	37.5	4	17.33 ± 0.57^*b*^	2.342	9.375	4	13.33 ± 0.57^*a*^	0.011	3
*P. aeruginosa* ATCC 27853	16 ± 2^*a*^	9.375	18.75	2	18.33 ± 1.52^*a*^	2.342	9.375	4	22.66 ± 0.57^*b*^	0.011	1.5

Yeasts	IZ^*∗*^	MIC	MFC*∗*^*∗*^	MFC/MIC ratio	IZ	MIC	MFC	MFC/MIC ratio	Amphotericin B		
									IZ	MIC	MFC

*Candida albicans* ATCC 2019	15 ± 1^*a*^	9.375	37.5	4	14.33 ± 0.57^*a*^	9.375	37.5	4	14.66 ± 0.57^*a*^	0.024	0.781
*Candida parapsilosis* ATCC 22019	14 ± 1^*b*^	9.375	37.5	4	15 ± 1^*b*^	9.375	37.5	4	10.33 ± 0.57^*a*^	0.195	0.39
*Candida krusei* ATCC 6258	17.66 ± 1.52^*b*^	9.375	37.5	4	10 ± 1^*a*^	9.375	18.75	2	12 ± 0 ^*a*^	0.097	0.195
*Candida tropicalis* ATCC 06-085	17 ± 1^*c*^	9.375	37.5	4	15 ± 1^*b*^	9.375	37.5	4	6 ± 0^*a*^	0.39	0.25

The diameter of the disc is 6 mm. The letters (a–c) indicate a significant difference between the different inhibition zones according to the Duncan test (*p* < 0.05). MIC: minimal inhibitory concentration expressed as mg/ml; MBC: minimal bactericidal concentration expressed as mg/ml; MFC: minimal fungicidal concentration expressed as mg/ml.

The article "Phytochemical Analysis, Antioxidant, Antimicrobial, and Anti-Swarming Properties of Hibiscus sabdariffa L. Calyx Extracts: In Vitro and In Silico Modelling Approaches" was published in 2022. Journal: Evid Based Complement Alternat Med.

**Table 4:** Determination of the MIC and MFC values of the different extracts tested on seven fungal strains (expressed in mg/mL).

Strains tested	*H. sabdariffa* methanolic extract	*H. sabdariffa* aqueous extract		
	MIC^*∗*^	MFC^*∗∗*^	MIC	MFC
*Aspergillus niger* DSM 63263	75	150	5	150
*Fusarium oxysporum*	150	>150	5	>150
*Penicillium expansum* DSM 1994	150	>150	5	>150
*Penicillium citrinum* DSM 1997	150	>150	5	>150
*Penicillium simplicissimum* DSM 1097	75	>150	5	>150
*Aspergillus versicolor* DSM 1993	150	>150	5	>150
*Aspergillus niger*	150	150	5	150

MIC: minimal inhibitory concentration (mg/ml); MFC: minimal fungicidal concentration (mg/ml).

**Table 5:** Comparative analysis of the results for the antioxidant activities obtained by DPPH, FRAP, and ABTS tests as compared to ascorbic acid.

*H. sabdariffa*	DPPH IC_50_ (mg/mL)	ABTS EC_50_ (mg/mL)	FRAP EC_50_ (mg/mL)
Methanolic extract	2.793 ± 0.044	2.082 ± 0.035	0.676 ± 0.026
Aqueous extract	2.471 ± 0.024	1.918 ± 0.060	0.578 ± 0.016
Ascorbic acid	0.022 ± 0.00058	0.0209 ± 0.0016	0.09 ± 0.007

**Table 6:** Evaluation of the anti-swarming activity of aqueous and methanolic extracts from *H. sabdariffa* against *P. aeruginosa* PAO1.

Mean diameter ± SD (mm)	Concentration of extracts in (mg/ml)					Standard
	**0.5**	**1**	**2.5**	**5**	**10**	
Aqueous extract	2.7 ± 0.25	1.2 ± 0.25	0	0	0	10.6 ± 0.57
Methanolic extract	9.6 ± 1.52	8.3 ± 0.57	0	0	0	9.5 ± 0.25

**Table 7:** Binding energy, conventional hydrogen bonds, and the closest interacting residues of 1JIJ, 2QZW, and 2UVO for TyrRS from *S. aureus*, the aspartic proteinase from *Candida albicans,* and the wheat germ agglutinin in complex with N-acetyl-D-glucosamine, respectively.

No.	Affinity (Kcal/mol)	Conventional H-bonds	Closest interacting residues	Distance to closest interacting residue (Å)
TyrRS from *S. aureus* (PDB ID: 1JIJ)				
1	−7.1	11	**Lys** ^**84**^ **, Arg** ^**88**^ **, Arg** ^**88**^ **, Tyr** ^**170**^ **, Gln** ^**174**^ **, Gln** ^**196**^ **, Asp** ^**80**^ **, Gly** ^**38**^ **, Gln** ^**196**^ **, Asp** ^**80**^ **, Gln** ^**196**^	Asp^80^ (2.25)
2	−9.1	7	**Lys** ^**84**^ **, Lys** ^**84**^ **, Asn** ^**124**^ **, Asp** ^**195**^ **, Asp** ^**177**^ **, Gln** ^**174**^ **, Gln** ^**190**^	Gln^174^ (1.92)
3	−9.1	6	**Cys** ^**37**^ **, Asp** ^**40**^ **, Thr** ^**75**^ **, Tyr** ^**170**^ **, Thr** ^**75**^ **, Asp** ^**195**^, Ala^39^, Gly^192^, Leu^70^	Thr^75^ (2.20)
4	−8.6	5	**Asp** ^**40**^ **, Gly** ^**193**^ **, Asp** ^**177**^ **, Gly** ^**38**^ **, Asp** ^**195**^, Ala^39^, Gly^192^, Leu^70^	Asp^195^ (2.09)
5	−8.9	8	**Gly** ^**38**^ **, Asp** ^**80**^ **, Arg** ^**88**^ **, Arg** ^**88**^ **, Gly** ^**193**^ **, Val** ^**191**^ **, Gln** ^**174**^ **, Asp** ^**40**^, Ala^39^, Lys^84^, Asp^195^, Asp^195^, His^50^, His^50^, Pro^53^	Arg^88^ (1.82)
6	−9.6	6	**Tyr** ^**36**^ **, Gln** ^**190**^ **, Asp** ^**177**^ **, Asp** ^**40**^ **, Thr** ^**75**^ **, Asp** ^**40**^, Ala^39^, Asp^195^, Ala^39^, Ala^39^	Thr^75^ (1.87)
7	−8.2	7	**Lys** ^**84**^ **, Arg** ^**88**^ **, Tyr** ^**170**^ **, Gln** ^**174**^ **, Gly** ^**193**^ **, Gln** ^**196**^ **, Asp** ^**40**^, Cys^37^, His^50^, His^50^, Asp^195^, Asp^195^, Asp^80^, Pro^53^, His^50^, Phe^54^, Cys^37^	Tyr^170^ (1.57)
8	−8.8	11	**Asp** ^**40**^ **, Asn** ^**124**^ **, Gln** ^**174**^ **, Gln** ^**174**^ **, Gly** ^**193**^ **, Gln** ^**196**^ **, Asp** ^**177**^ **, Asp** ^**177**^ **, Asp** ^**195**^ **, Gly** ^**49**^ **, Gln** ^**190**^, His^50^, Gly^38^, Asp^40^, His^50^, Ala^39^, Ala^39^	Asp^40^ (1.60)
9	−8.3	9	**Cys** ^**37**^ **, Lys** ^**84**^ **, Lys** ^**84**^ **, Arg** ^**88**^ **, Arg** ^**88**^ **, Gln** ^**174**^ **, Asp** ^**40**^ **, Thr** ^**75**^ **, Asp** ^**40**^, Asp^40^, Asp^195^, Asp^195^, Cys^37^, His^50^, Tyr^36^, Ala^39^, Pro^53^	Lys^84^ (2.24)
10	−9.4	4	**Lys** ^**84**^ **, Lys** ^**84**^ **, Arg** ^**88**^ **, Asp** ^**177**^, Asp^80^, Asp^80^, Leu^70^	Lys^84^ (2.50)

*Aspartic proteinase from Candia albicans (PDB ID: 2QZW)*				

1	−5.2	5	**Asp** ^**218**^ **, Thr** ^**221**^ **, Asp** ^**218**^ **, Asp** ^**218**^ **, Asp** ^**86**^	Asp^86^ (2.13)
2	−6.2	6	**Gly** ^**85**^ **, Asn** ^**131**^ **, Arg** ^**192**^ **, Arg** ^**195**^ **, Thr** ^**221**^ **, Glu** ^**193**^	Asn^131^ (2.01)
3	−5.7	5	**Asn** ^**131**^ **, Arg** ^**195**^ **, Thr** ^**221**^ **, Asp** ^**32**^ **, Gly** ^**34**^	Asp^32^ (2.14)
4	−4.1	2	**Gly** ^**220**^ **, Glu** ^**193**^, Asp^86^, Asp^218^, Ile^30^, Ile^123^	Glu^193^ (2.42)
5	−0.3	3	**Ser** ^**35**^ **, Gly** ^**220**^ **, Gly** ^**220**^, Asp^86^, Asp^218^, Asp^218^, Gly^85^, Tyr^84^, Leu^216^, Ala^335^	Gly^220^ (1.87)
6	−7.8	2	**Arg** ^**195**^ **, Asp** ^**86**^, Asp^86^, Asp^218^, Asp^218^, Gly^85^, Leu^216^, Ala^335^	Asp^86^ (2.60)
7	26.3	4	Asp^86^, Asp^218^, **Leu**^**217**^**, Thr**^**33**^**, Ser**^**35**^**, Thr**^**221**^, Arg^192^, Glu^193^, Leu^216^, Leu^216^	Thr^221^ (1.47)
8	32.6	6	**Gly** ^**34**^ **, Gly** ^**34**^ **, Gly** ^**220**^ **, Gly** ^**220**^ **, Glu** ^**193**^ **, Ala** ^**303**^, Gly^220^, Asp^218^, Asp^218^, Thr^221^, Ile^305^, Leu^216^, Ala^303^, Ile^305^, Ala^335^	Gly^220^ (2.47)
9	31.2	2	Glu^193^, Asp^218^, Glu^193^, Asp^218^, **Ser**^**35**^**, Gly**^**85**^, Ser^35^, Thr^221^, Ser^336^, Asp^32^, Asp^32^, Ile^123^, Tyr^84^, Tyr^84^, Ile^123^, Ile^30^	Ser^35^ (1.66)
10	−7.5	4	**Gly** ^**220**^ **, Gly** ^**34**^ **, Glu** ^**193**^ **, Ala** ^**303**^, Asp^218^, Asp^218^, Leu^216^, Ala^303^, Ala^335^	Glu^193^ (2.10)

Wheat germ agglutinin (PDB ID: 2UVO)				

1	−5.1	8	**Arg** ^**45**^ **, Arg** ^**45**^ **, Gln** ^**49**^ **, Tyr** ^**66**^ **, NAG** ^**1174**^ **, Tyr** ^**64**^ **, NDG** ^**1173**^ **, NA** ^**1174**^	Tyr^64^ (2.32)
2	3.2	6	**Cys** ^**55**^ **, Asn** ^**58**^ **, Asn** ^**58**^ **, Gln** ^**59**^ **, Gln** ^**59**^ **, Gln** ^**59**^, Pro^82^, Ile^87^, Phe^69^, Pro^82^, Leu^102^	Gln^59^ (1.72)
3	−1.1	5	**Ser** ^**43**^ **, Arg** ^**45**^ **, NDG** ^**1173**^ **, NAG** ^**1174**^ **, Ser** ^**43**^, Thr^42^, Ser^43^, Tyr^66^	Ser^43^ (1.92)
4	−4.8	1	**Tyr** ^**66**^, NAG^1174^, Tyr^64^	Tyr^66^ (2.15)
5	4.8	3	**Cys** ^**55**^ **, Gln** ^**59**^ **, Cys** ^**55**^, Leu^102^, Gly^81^, Phe^69^, Pro^99^/Asn^100^, Pro^82^, Pro^99^, Leu^102^, Pro^82^, Ile^87^, Pro^99^	Cys^55^ (2.00)
6	−6.9	2	**Arg** ^**45**^ **, Tyr** ^**64**^, Tyr^64^, Tyr^64^, Tyr^66^	Tyr^64^ (1.74)
7	15.4	6	**Gly** ^**70**^ **, Gly** ^**52**^ **, Gln** ^**59**^ **, Cys** ^**83**^ **, Ala** ^**85**^ **, Cys** ^**83**^, Gly^81^, Cys^110^, Cys^83^, Cys^55^, Cys^61^, Asn^100^, Gln^79^/Gly^80^, Pro^82^, Cys^60^, Cys^74^, Pro^99^, Pro^99^	Cys^83^ (1.75)
8	19.8	6	**Ser** ^**43**^ **, Ser** ^**43**^ **, Lys** ^**44**^ **, Lys** ^**44**^ **, Gly** ^**38**^ **, Gln** ^**59**^, Thr^42^, Lys^44^, Gly^38^, Cys^103^, Cys^117^, Gly^113^/Ser^114^, Gly^113^/Ser^114^, Lys^44^, Cys^55^, Cys^67^, Cys^117^, Leu^112^, Ala^125^, Ala^39^	Lys^44^ (2.15)
9	16	6	**Gly** ^**81**^ **, Ile** ^**87**^ **, Asn** ^**100**^ **, Asn** ^**58**^ **, Cys** ^**110**^ **, Gly** ^**52**^, Gly^47^, Gly^80^, Gly^81^, Asn^100^, Ala^53^, Gln^79^, Phe^69^, Phe^69^, Phe^69^, Pro^82^, Ile^87^, Pro^82^, Ile^87^, Pro^82^, Leu^102^	Asn^58^ (1.67)
10	6.3	3	**Arg** ^**45**^ **, Tyr** ^**66**^ **, NAG** ^**1174**^, Tyr^64^	Tyr^66^ (1.92)

The article "Phytochemical Analysis, Antioxidant, Antimicrobial, and Anti-Swarming Properties of Hibiscus sabdariffa L. Calyx Extracts: In Vitro and In Silico Modelling Approaches" was published in 2022. Journal: Evid Based Complement Alternat Med.

## Data Availability

All data generated or analyzed during this study are included in this article.
